RETRACTED

# Effect Analysis of Nursing Method Based on Stratified Emergency Knowledge in Emergency Myocardial Infarction

**DOI:** 10.1155/2022/3505228

**Published:** 2022-09-30

**Authors:** Junxia Yu, Jie Mu

**Affiliations:** ^1^Kaifeng Central Hospital, Kaifeng, 475000 Henan, China; ^2^Kaifeng Vocational College of Culture and Art, Kaifeng, 475000 Henan, China

## Abstract

First aid is to give immediate first aid to patients who have suffered accidental injuries or sudden diseases before the emergency medical personnel arrive at the scene or are sent to the hospital for treatment; myocardial infarction is a severe and emergency of coronary heart disease. It is often because of coronary atherosclerosis, plaque rupture, bleeding, or thrombosis, which leads to the acute and complete occlusion of the coronary arteries and acute necrosis of the myocardium. This article aims to investigate the effectiveness of a stratified emergency care team assisted by multidisciplinary first aid knowledge in acute myocardial infarction first aid, hoping to reduce the probability of acute myocardial infarction through first aid and nursing care. Business process reengineering is a management idea that reached its heyday in the 1990s and is usually defined as achieving workflow and productivity through the reorganization and optimization of corporate strategies, value-added operational processes, and the systems, policies, organizations, and structures that support them. This article first outlines the concepts and steps of medical image registration, analyzes the characteristics of current medical image registration methods, and uses the two most commonly used medical registration methods today; in this study, the BPR theory was used to construct the AMI emergency care process in the hospital, which effectively reduced the emergency delay time of AMI patients, improved the patient's emergency response, and increased the efficiency of emergency nurses' rescue work. The experimental results in this paper show that the sensitivities of the first four groups of ST↑III > II, ST ↓ aVL > I, STV3 ↓ /STIII↑≤1.2, STI ↓ ≥0.05 mV are 82.1%, 80%, 75.3%, and 60.3%, respectively. Their sensitivities are relatively close, both are greater than 50%; among them, ST↑III > II has the highest sensitivity, which is 80%. In terms of specificity, ST↑III > II, ST ↓ aVL > I, STV3 ↓ /STIII↑≤1.2, and STI ↓ ≥0.05 mV were 82.1%, 89.2%, 82.7%, and 65.2%, respectively. ST ↓ ≥0.05 mV has the lowest specificity, and ST ↓ aVL > I has the highest specificity.

## 1. Introduction

Myocardial infarction is one of the most fatal and disabling diseases with the highest risk; so, its greatest harm can be said to be death. Myocardial infarction, also called myocardial infarction, is mainly caused by partial necrosis of myocardium due to ischemia caused by interruption of blood flow. Due to the continuous development of the economy, the pace of life is getting faster and faster, and the pressure of life is getting heavier. Overwork has become a common phenomenon nowadays. Excessive exertion brings about an increase in myocardial oxygen consumption, plaque rupture, and myocardial infarction. In recent years, there have been more and more cases of myocardial infarction, and the age of the onset group is getting younger and younger. The continuous enhancement of these characteristics requires that we urgently need to find an effective way to reduce the mortality rate of acute myocardial infarction. With the improvement of people's living standards and people's attention to improving the quality of life, the mastery of first aid knowledge has become a new trend at the moment. If the patient can be treated with emergency treatment in time, this can save the patient's life to a large extent and delay the deterioration of the condition. In particular, for sudden heart diseases such as acute myocardial infarction, if effective first aid can be given in time, doctors can be left with time for rescue. Therefore, combining the stratified emergency care team assisted by the knowledge of the department and the acute myocardial infarction first aid will have a huge effect on patients with acute myocardial infarction, thereby reducing the mortality rate. Myocardial infarction is one of the most common diseases that endanger human health. The World Health Organization pointed out that in the past few decades, the understanding of myocardial infarction has been continuously deepened, and the mortality rate under treatment has decreased significantly, with the mortality rate of hospitalized patients reaching 11.9%. Although some progress has been made in myocardial infarction in recent years, many detection techniques are only adapted to a certain stage. Combining the stratified first-aid care team assisted by the knowledge of departmental first aid and acute myocardial infarction first aid is of great practical significance for improving survival and treatment. Advances in diagnostic techniques, its electrocardiogram, are currently developed from surface electrocardiograms to intracardiac electrophysiological electrograms. Intravascular ultrasonography can also be done to determine the type of thrombus and the condition of the lesion.

RETRACTED

The implementation of full-time stratified nursing can effectively improve the quality of nursing. After systematic training, the nursing staff can effectively improve their first aid skills and can accurately judge the changes in the condition and implement rescue measures. Although some progress has been made in myocardial infarction in recent years, many detection techniques are only adapted to a certain stage. Therefore, the combination of the stratified emergency care team assisted by the knowledge of departmental first aid in the first aid of acute myocardial infarction is still the current research focus. Noris et al. studied isolated spontaneous platelet aggregation (SPA) in platelet-rich plasma from 37 patients with acute myocardial infarction. It occurs in subjects who receive heparin after streptokinase therapy and rarely occurs in patients who have not received streptokinase or heparin therapy and in patients who have received streptokinase therapy alone. Research on patients receiving heparin therapy for deep vein thrombosis suggests that SPA may come from adenosine diphosphate released by platelets during sample processing. Therefore, Noris P suggested that heparin infusion may promote platelet activation in vitro, and this mechanism is effective in patients with acute myocardial infarction receiving thrombolytic therapy [1]. Eicher et al. expanded these RNA-seq studies by completing RNA-seq in platelets from 32 patients with acute myocardial infarction (MI). The transcripts in platelets are mainly produced in precursor megakaryocytes, but they still maintain physiological activity when platelets translate RNA and regulate protein/RNA levels. The goal of this experiment is to use a group of patients with acute MI to characterize the platelet transcriptome. And the gene expression and platelet aggregation measurement and ST segment elevation MI (STEMI) (*n* = 16) and non-STEMI (NSTEMI) (*n* = 16) subtypes were associated. Similar to other studies, 9565 expressed transcripts were detected, including several known platelet-rich markers (such as PPBP and OST4). RNA-seq data is closely related to independently determined platelet expression data. It also shows the enrichment of platelet-related pathways (such as wound response, hemostasis, and platelet activation), as well as actin-related and posttranscriptional processes [2]. Shah et al. proposed to assess the association between acute myocardial infarction and hospitalized survivors' postdischarge mortality and all-cause hospitalization. He also included AMI patients 65 ≥ years old from the ACTION Registry-GWTG (Acute Coronary Artery Treatment and Intervention Results Network Registration-Follow Guidelines). These patients survived the hospitalization, and he linked these patients with medical insurance claim data. He uses a proportional hazard model to test the association between acute myocardial infarction and outcome and adjusts it according to patient and hospital characteristics. Report the hazard ratio (HR) in the early period (1 to 60 days) and late period (61 to 365 days) after discharge. Among 112,668 survivors of AMI, 5% developed acute myocardial infarction during hospitalization. Patients with acute myocardial infarction have significantly higher mortality rates for 60 days (9.6% vs. 5.5%) and 1 year (22.4% vs. 16.7%) [3]. Avau et al. described a protocol for a cluster randomized controlled trial. The trial will investigate the impact of using simulated patients on basic first aid training for nonprofessionals on their knowledge, skills, and self-efficacy. The study is that the use of patient simulators during basic first aid training does not lead to statistically significant changes in knowledge, skills, and self-efficacy on the topic of first aid using patient simulators. Another option is to use simulated patients during training that affects knowledge, skills, and self-efficacy. The experiment proved that teaching first aid knowledge to nonprofessionals is a cost-effective way to improve public health [4]. Qy et al. uses a questionnaire survey to investigate first aid knowledge and treatment options for children with small burns. The effective rate of the questionnaire is 99.4% (5814/5850). It was found that 17.8% (1,036/5814) and 48.9% (2841/5814) had chosen folk remedies and daily necessities, respectively, and 39.8% (2,312/5814) of nursing staff knew all standard burn first aid measures. In addition, the proportion of caregivers with a bachelor's degree in understanding the five indicators is significantly higher than that of other educational backgrounds. Caregivers lack first aid knowledge of small burns in children. Only a few nurses know all five standard first aid measures for managing small burns [5]. Zhang et al. investigated the association between short-term PM exposure and emergency department visits (EDV) for AMI, ST-segment elevation myocardial infarction (STEMI), and non-ST-segment elevation myocardial infarction (NSTEMI). The experiment conducted a case-crossover study on 2749 AMI patients who were hospitalized in Anzhen Hospital in Chaoyang District in 2014. Meteorological and air pollution data were collected during this period. The experiment uses a time-layered case crossover design with a lag model. Adjusting according to meteorological conditions and/or other gaseous pollutants to estimate the EDV risk of AMI, STEMI, and NSTEMI, a stratified analysis was performed by gender, age, season, and comorbidities to check for potential impact corrections. It was found that every 10 *μ*g/m^3^ increase in PM2.5 concentration (with a lag of 1 day) is associated with an increase in the risk of EDV [6]. Zhang et al. studied the effect of a 12-lead ECG real-time remote transmission system on the door-to-balloon time of athletes with ST-segment elevation myocardial infarction. Sixty athletes with chest pain diagnosed with ST-segment elevation myocardial infarction (STEMI) were randomly divided into group A (*n* = 35) and group B (*n* = 25). The 12-lead ECG timing teletransmission system was sent to the chest pain center before the patients in group A were transferred to the hospital, while the patients in group B did not. The median time from door to balloon in group A was significantly shorter than that in group B (38 minutes vs. 94 minutes, *p* < 0.05). The median length of hospital stay in group A was significantly shorter (5 days vs. 7 days, *p* < 0.01). Experiments have proved that the 12-lead ECG real-time remote transmission system is beneficial to the prehospital diagnosis of STEMI [7]. Although these theories have a certain degree of discussion on first aid knowledge and acute myocardial infarction, due to the limitations of conditions, they still cannot be implemented in many aspects.

RETRACTED

At present, most of the research on the emergency system is a single center; in short, it is a research on a regional collaborative rapid treatment system with a PCI hospital as the core [8]. Therefore, there has not been a multicenter study of the *N* + *n* regional collaborative rapid treatment system established by multiple PCI hospitals as the core. In this study, many hospitals are covered, and the geographical scope is very broad, allowing a more comprehensive analysis of acute myocardial infarction.

## 2. The Effect Investigation Method of the Stratified Emergency Care Team Assisted by Multidisciplinary First Aid Knowledge in the First Aid of Acute Myocardial Infarction

### 2.1. Acute Myocardial Infarction

With the continuous development of the economy and the increasing aging, cardiovascular disease has become one of the major causes of mortality. According to WHO statistics, there are currently about 500 million people suffering from cardiovascular diseases in the world, while more than 300 million people in China [9]. This data is sufficient to show that cardiovascular disease has become the main cause of resident mortality, smoking, obesity, and diabetes which are the main causes of cardiovascular disease [10]. In cardiovascular diseases, ischemic heart disease is a common cause of myocardial infarction. However, according to data, the mortality rate of myocardial infarction due to ischemia is declining in Western Europe. Although the overall data is declining, the mortality rate is still not to be underestimated. According to survey data, the incidence of myocardial infarction in women is lower than that in men, and the age of onset is older than that in men, but myocardial infarction is still a major cause of female mortality [11, 12]. Myocardial infarction is a blockage of the coronary arteries, resulting in myocardial ischemic necrosis caused by insufficient blood supply to the myocardium. When patients suffer from acute coronary occlusion, the heart muscle will be necrotic due to lack of blood supply.  Figure 1 is a schematic diagram of myocardial infarction:

Acute myocardial infarction is an acute myocardial ischemic heart disease, including ST-segment elevation myocardial infarction and non-ST-segment elevation myocardial infarction [13]. The main reason is that the arteries are ruptured or eroded, so that the thrombotic substances inside the plaque appear in the blood, which causes the activation of platelets in the plaque to form different types of thrombus. If the thrombosis completely occludes the coronary artery, we call it an infarct-related artery; if the thrombosis does not completely occlude the coronary artery, we call it a criminal vessel. According to research, the deterioration of plaque is related to inflammation, immune response, and thrombosis, but plaque rupture is the main cause of acute myocardial infarction [14, 15]. There are many risk markers in epidemics. According to research, if the risk markers are intervened, the mortality of acute myocardial infarction can be reduced. Currently recognized dangerous substances in the medical profession include high blood pressure, diabetes, obesity, and family history. If the abovementioned dangers can be avoided, coupled with the scientific management of blood sugar and blood pressure, the mortality rate of acute myocardial infarction can be greatly reduced. Acute myocardial infarction is a potentially very harmful disease. General treatment methods include oxygen inhalation and bed rest. It can also be treated with anticoagulation and lipid-lowering drugs or coronary revascularization [16]. Regardless of the method used, the fundamental purpose is to restore the blood perfusion of the myocardium and to save the dying myocardium and maintain normal heart function. As a result of years of research on acute myocardial fibers, scholars have found that reasonable diet, physical exercise, quitting smoking and drinking, and regulating blood pressure can effectively prevent the occurrence of acute myocardial infarction to a certain extent. However, the acute myocardial infarction has been diagnosed, and active treatment is needed to prevent it from turning into a worse condition [17, 18].

RETRACTED

### 2.2. Image Detection of Acute Myocardial Infarction

In order to obtain the image information of myocardial infarction, data collection of the entire image is required. Connect each point of the image to make the diagnosis information more accurate [19]. Define the function expression of the digital image as

(1) $$\begin{array}{c} g\left(a,b\right)=\left[\begin{array}{c} g\left(1,1\right)g\left(1,2\right)\cdots g\left(1,n\right)\\ g\left(1,2\right)g\left(2,2\right)\cdots g\left(2,n\right)\\ \vdots \\ g\left(n,1\right)g\left(n,2\right)g\left(n,n\right) \end{array}\right] \end{array}$$

where (*a*, *b*) represents the floating image point.

(2) $$\begin{array}{c} S_{g}\left(a,b\right)=y\left(S_{g}\left(g\left(a,b\right)\right)\right). \end{array}$$

*S*_*g*_(*a*, *b*) represents the gray value of the target point, *g* represents the displacement function of the image, and *y* represents the change function of the pixel value. The premise of pixel value transformation is spatial transformation, but this transformation does not occur under any circumstances.  Figure 2 is a schematic diagram of image space conversion. When it changes, the function expression can be described as

(3) $$\begin{array}{c} S_{g}\left(a,b\right)=S_{g}\left(g\left(a,b\right)\right). \end{array}$$

The main job of parameter conversion is to determine the coincidence point. Coincidence point refers to a large point (or control point of each level) that has coordinates of two coordinate systems at the same time. In the formal image space conversion, we need to determine the conversion process, especially the parameter conversion. Find the corresponding relationship between the parameters, and the main operation process is shown in Figure 3:

Projection transformation is the process of transforming the coordinates of one map projection point into the coordinates of another map projection point. Research the theory and method of coordinate transformation of projected point. The transformation of the search space includes global transformation, local transformation, and semilocal transformation. The semilocal transformation can be divided into rigid body transformation, affine transformation, projection transformation, and nonlinear transformation [20, 21]. The distance between the two points before and after transformation remains unchanged, which is called rigid body transformation. Rigid body transformation can be decomposed into translation transformation, rotation transformation, and inversion (mirror) transformation. Rigid body transformation is a combination of rotation and translation, representing the rotation angle between the target image and the vertical translation. The function expression is as follows:

(4) $$\begin{array}{c} \left[\begin{array}{c} a^{\prime }\\ b^{\prime }\\ 1 \end{array}\right]=\left[\begin{array}{ccc} \cos\alpha & ‐\sin\alpha & {\text{Q}}_{\text{a}}\\ \sin\alpha & \cos\alpha & {\text{Q}}_{\text{b}}\\ 0 & 0 & 1 \end{array}\right]\left[\begin{array}{c} a\\ b\\ 1 \end{array}\right]. \end{array}$$

Affine transformation, also known as affine mapping, means that in geometry, a vector space is transformed into another vector space by performing a linear transformation followed by a translation. *α* represents the strain of the rigid body transformation, *Q*_*a*_ represents the rotation angle, and *Q*_*b*_ represents the displacement that occurs in the horizontal and vertical directions.

RETRACTED

The affine transformation is converted from the rigid body transformation. It adds scaling and miscutting on the basis of rotation and translation. All in all, two degrees of freedom are added on the basis of rigid body transformation [22]. The function expression is as follows:

(5) $$\begin{array}{c} \left[\begin{array}{c} a^{\prime }\\ b^{\prime }\\ 1 \end{array}\right]=\left[\begin{array}{ccc} s_{11} & {\text{s}}_{12} & {\text{Q}}_{\text{a}}\\ s_{21} & s_{22} & {\text{Q}}_{\text{b}}\\ 0 & 0 & 1 \end{array}\right]\left[\begin{array}{c} a\\ b\\ 1 \end{array}\right]. \end{array}$$

*s*_11_, *s*_12_, *s*_21_, *s*_22_, *Q*_*a*_, *Q*_*b*_ represents the parameter change point, which can be determined by three points on any straight line.

The biggest feature of projection transformation is that it can convert straight lines into straight lines, but it cannot keep it balanced. This application is more common in registration between multi-dimensional images [23]. The function expression is as follows:

(6) $$\begin{array}{c} \left[\begin{array}{c} a^{\prime }\\ b^{\prime }\\ c^{\prime } \end{array}\right]=\left[\begin{array}{ccc} s_{11} & s_{12} & s_{13}\\ s_{21} & s_{22} & s_{23}\\ s_{31} & s_{32} & s_{33} \end{array}\right]. \end{array}$$

The degrees of freedom of projection transformation include rotation, shearing, scaling, and translation, which can be determined by any three points that are not collinear. Linear transformation uses polynomial functions to map straight lines into straight lines [24]. Nonlinear transformation can control the smoothness of the deformation, which is suitable for the image subject of global geometric deformation.  Figure 4 is a schematic diagram of the four transformations:

The thin plate spline is obtained by the researchers through the results of scattered data, and it is also one of the most used methods in medical imaging. Thin-plate spline interpolation is a kind of interpolation method and is a commonly used 2D interpolation method. The function expression is as follows:

(7) $$\begin{array}{c} g\left(o,p\right)=c_{0}+c_{1}o+c_{2}p+\overset{m}{\underset{j=1}{\sum }}Q_{j}t_{j}^{2}\ln t_{j}^{2}. \end{array}$$

Among them,

(8) $$\begin{array}{c} t^{2}={\left(o-o_{j}\right)}^{2}+{\left(p-p_{j}\right)}^{2}+e^{2}. \end{array}$$

*e* ^2^ represents the stiffness parameter. When *e*^2^ is close to zero, the load is close to the point load. When *e*^2^ shows an increasing trend, the load becomes smoother.

(9) $$\begin{array}{c} \overset{m}{\underset{j=1}{\sum }}Q_{j}=\overset{m}{\underset{j=1}{\sum }}Q_{j}o_{j}=\overset{m}{\underset{j=1}{\sum }}Q_{j}p_{j}=0. \end{array}$$

Loads refer to external forces and other factors that cause internal forces and deformations of structures or components or conventionally refer to various direct actions that are applied to engineering structures to produce effects on engineering structures or components. When the load is zero, the thin plate is in a stable state, so that the surface will not rotate. Solve the equations to get the coefficients, and the thin plate can undergo arbitrary deformation at the mark definition point [25].

(10) $$\begin{array}{c} A=\left\{\left(A,B,C\right)\left|0\leq a\leq A,0\leq b\leq B,0\leq c\leq C\right.\right\}. \end{array}$$

*A* represents the area of the image.

(11) $$\begin{array}{c} \overset{⟶}{f}\left(a,b,c\right)=\overset{3}{\underset{k=0}{\sum }}\overset{3}{\underset{h=0}{\sum }}\overset{3}{\underset{r=0}{\sum }}S_{k}\left(f\right)S_{h}\left(d\right)S_{r}\left(l\right). \end{array}$$

Among them, $\overset{⟶}{f}$ represents the displacement field, and the distance between them is *V*.

(12) $$\begin{array}{c} S_{0}\left(f\right)=\frac{{\left(1-f\right)}^{3}}{6},\\ S_{1}\left(f\right)=\frac{3f^{3}-6f^{2}+7}{6},\\ S_{2}\left(f\right)=\frac{-3f^{3}+3f^{2}+3f+1}{6},\\ S_{3}\left(f\right)=\frac{f^{3}}{6}, \end{array}$$

where *S*_*n*_ represents the basis function of the *n*-th *S*-spline.

RETRACTED

In information theory, mutual information can be used to express the size and relevance of the amount of information in the system. The function expression is as follows:

(13) $$\begin{array}{c} W\left(C,D\right)=\underset{c,d}{\sum }E_{cd}\left(c,d\right)\log_{2}\frac{E_{cd}\left(c,d\right)}{E_{C}\left(c\right)*E_{D}\left(d\right)}. \end{array}$$

Among them, *C* and *D* represent two images, *E*_*c*_, *E*_*d*_ represents the probability distribution, and *E*_*cd*_ represents the joint probability distribution.

(14) $$\begin{array}{c} U=\frac{\sum_{\left(x,y\right)\in Z}\left(C\left(x,y\right)-\bar{C}\right)\left(D\left(x,y\right)-\bar{D}\right)}{\sqrt{\sum_{\left(x,y\right)\in z}{\left(C\left(x,y\right)-\bar{C}\right)}^{2}\sum_{\left(x,y\right)\in z}{\left(D\left(x,y\right)-\bar{D}\right)}^{2}}}. \end{array}$$

Among them, *U* represents normalized information, *C* and *D* represent two images, and *C*(*x*, *y*), *D*(*x*, *y*) represents the gray value of the image at point (*x*, *y*).

(15) LC=−∑ceccloge2cc,LD=−∑deddlog2edd,LC,D=−∑c,decdc,dlog2ecdc,d,P=LC+LDLCD.

Among them, *c* ∈ *C*, *d* ∈ *D*, *e*_*c*_(*c*), *e*_*d*_(*d*) represents the independent distribution probability of the system, *e*_*cd*_ represents the joint distribution probability, *L*(*C*), *L*(*D*) represents the entropy of C and D, and *L*(*C*, *D*) represents the joint entropy.

### 2.3. First Aid Knowledge

According to the survey of relevant data, if the heart stops beating within 4 minutes and effective first aid can be obtained, the patient has a half chance of surviving. Once rescue is carried out after 10 minutes, the probability of survival of the patient is very small, less than 1% [26]. Therefore, the mastery of first aid knowledge will produce great value in practical applications. However, the popularization of first aid knowledge in China is relatively late, and the awareness of first aid is still relatively weak. Most people regard cardiopulmonary resuscitation as a very difficult operation [27]. In fact, emergency medicine is very practical, and once the operation is successful, it is very difficult to save a life. In the actual medical process, doctors rarely have the opportunity to perform emergency operations unless the patient is in the hospital when the disease occurs. Therefore, whether it is a doctor or an ordinary person, it is essential to master first aid knowledge [28].

At present, the teaching of first aid knowledge in China is basically based on textbooks. However, these teaching methods cannot simulate the real situation and cannot create a sense of crisis in the first aid scene; so, the teaching effect is not very good [29]. The emergence of simulated first aid systems in recent years has effectively improved the shortcomings of human teaching. The system can simulate various patient disease states. It can produce corresponding changes through different first aid methods to detect the correctness of the first aid measures.  Figure 5 is a schematic diagram of the system structure.

The most common feature of patients with acute myocardial infarction is chest pain, and coronary stenting can effectively alleviate this condition. However, there are still many problems in the care of acute myocardial infarction in China. The common ones are unclear division of labor, chaotic emergency scenes, error-prone, and waste of resources. Through literature research, the nursing process in medical institutions in Western countries is divided into three categories: cardiovascular care, chest pain emergency care, and emergency care. It does not treat acute myocardial infarction as a major prescribed nursing process. In the first aid part of the hospital management process, the value specifies information such as the emergency environment, patient evaluation, and clinical records [30]. However, these first aid procedures are not detailed, only the framework. Even in the first aid guide, the focus is on operations such as cardio-cerebrovascular diseases and cardiopulmonary resuscitation, and there is too much discussion on acute myocardial infarction. Chinese chest pain center is the largest acute myocardial infarction emergency system, and the emergency process has been carefully regulated during its overview. However, there are still many unreasonable points, such as responsibilities that cannot be implemented, nursing content is easy to repeat, and nursing procedures are too simple.

RETRACTED

Nursing of acute myocardial infarction is very important and affects the prognosis of patients. General routine nursing measures include observing the patient's condition, finding out the discomfort in time, and assisting the patient to take medicine, eat, drink water, and defecate. The current nursing process for acute myocardial infarction is still in the development stage. The subject of inquiry lacks pertinence, which is not much different from the ordinary nursing process, and the process is not detailed enough. For example, the establishment of full-time nurses in the emergency department and systematic training of nurses can improve the nursing ability of acute myocardial infarction, which indeed improves the nursing level of acute myocardial infarction to a certain extent, but the complete nursing process has not yet been implemented. In view of these conditions, it is not difficult to find that the current acute myocardial infarction care process lacks specificity and cannot adapt to acute myocardial infarction emergency care; nursing responsibilities cannot be fulfilled, reliance on experience is strong, and resources are wasted; the model is outdated and cannot keep up with the development of chest pain centers [31, 32].

## 3. The Effect Investigation Experiment of Stratified Emergency Nursing Team Assisted by Multidisciplinary First Aid Knowledge in the First Aid of Acute Myocardial Infarction

### 3.1. Research Objects

According to the definition of acute myocardial infarction, the subjects of this investigation need to have the following characteristics: myocardial loss or ventricular wall displacement phenomenon, abnormal troponin detection, presenting symptoms of acute myocardial ischemia, coronary angiography,; and coronary thrombosis [33]. The age, sex, blood pressure, symptoms, and treatment of patients with acute myocardial infarction were recorded, the patients with acute myocardial infarction were divided into two groups, and the effectiveness and expected status of the treatment between the two groups were compared.

RETRACTED

According to the data in Table 1, this experiment was mainly male and was divided into two groups for observation. The patients in the two groups were between 66and 67 years old, with 300 people in each group. During the recording of blood pressure, it was found that patients generally had hypertension symptoms, and diabetes was also very common. The number of people with a history of the disease was relatively small. In general, there was no significant difference between the two groups of patients.

### 3.2. Comparison of Treatment Time of Patients with Myocardial Infarction

According to the data in Table 2, the variables of this investigation include percutaneous coronary intervention and acute percutaneous coronary intervention, that is, total myocardial ischemia time, time from onset to arrival at the hospital gate, time from onset to first medical contact, and time from first medical contact to balloon expansion. According to the data, the number of patients undergoing percutaneous coronary intervention and acute percutaneous coronary intervention is not much different between the two groups. The total myocardial ischemia time of the second group was significantly higher than that of the first group, and the difference between the time from onset to the first medical contact between the two groups was very small; the time from first medical contact to balloon dilation of the second group was higher than that of the first group. In the comparison of the time from onset to arrival at the hospital gate, the first group was faster than the second group.

According to the data in Figure 6, the time difference between the patient's onset and the first medical contact is not obvious, which will not interfere much with subsequent treatment; there is a small gap between the time between the onset of the patient and the first medical contact between the two groups; the time difference between the patient's onset and arrival at the hospital is very small, faster than negligible; the total myocardial ischemia time of the first group was longer than that of the second group, but the difference was not obvious.

RETRACTED

### 3.3. Vascular Conditions in Patients with Myocardial Infarction

According to the data in Table 3, it is divided into four groups according to the blood vessels of coronary artery disease. In the ST-segment elevation myocardial infarction group, there were 1 case of coronary artery in good condition, 240 cases of single-vessel disease, 45 cases of double-vessel disease, and 7 cases of multivessel disease. In the non-ST segment elevation myocardial infarction group, there were 0 cases of coronary artery in good condition, 90 cases of single-vessel disease, 130 cases of double-vessel disease, and 40 cases of multivessel disease.

According to the data in Table 4, the sensitivity of the first four groups of ST↑III > II, ST ↓ aVL > I, STV3 ↓ /STIII↑≤1.2, and STI ↓ ≥0.05 mV are 82.1%, 80%, 75.3%, and 60.3%, respectively. They are relatively close, both are greater than 50%; among them, ST↑III > II has the highest sensitivity for prediction, which is 80%. In terms of specificity, ST↑III > II, ST ↓ aVL > I, STV3 ↓ /STIII↑≤1.2, and STI ↓ ≥0.05 mV were 82.1%, 89.2%, 82.7%, and 65.2%, respectively. ST ↓ ≥0.05 mV has the lowest specificity, and ST ↓ aVL > I has the highest specificity.

## 4. Investigation and Analysis of the Effect of Stratified Emergency Nursing Team Assisted by Multidisciplinary First Aid Knowledge in the First Aid of Acute Myocardial Infarction

### 4.1. Cardiac Function in Patients with Acute Myocardial Infarction

According to the data in Figure 7, there is no difference in the walking distance of the two groups of patients within 5 minutes before the experiment. After one month of intervention between the two groups of patients, although the difference between the experimental group and the control group has expanded to a certain extent, the difference is not obvious. After two months of intervention, the walking distance of the control group was 243 m, and the walking distance of the experimental group was 286 m. After three months of intervention, the walking distance of the control group was 250 m, the walking distance of the experimental group was 349 m, the walking distance gap gradually widened, and the recovery of the experimental group was significantly better than that of the control group.

In a controlled experiment on changes in left ventricular ejection fraction of patients with acute myocardial infarction, there was no significant difference between the two groups of patients before the intervention. After two months of intervention, no recovery advantage was seen. At the third month of the intervention, the ejection fraction of the control group was 51, while the ejection fraction of the experimental group was 64. The recovery status of the experimental group was significantly better than that of the control group.

RETRACTED

### 4.2. Comparison of Overall Treatment Effects

According to the data in Figure 8, in the overall treatment effect of the two groups of patients, 9 cases were cured in the control group, 3 cases were markedly effective, 2 cases were effective, and 6 cases were ineffective. In the experimental group, 17 cases were cured, 4 cases were markedly effective, 1 case was effective, and 4 cases were ineffective. The difference in the number of patients recovered between the two groups is very large, indicating that the recovery rate after professional care is better, and there are more patients with marked effects. Comparing the experimental group with the control group, there was no significant difference in the scores of the two groups before treatment. After treatment, the score of the control group was 4.4, while the score of the experimental group was only 2.2. The average score of the experimental group is 6.3, and the average score of the experimental group is 5.4. After treatment, the points of the experimental group decreased significantly compared with the control group, and the difference was large, indicating that the nursing of the treatment group had a better improvement effect.

Cardiac enzymes are a general term for a variety of enzymes present in the myocardium, including aspartate aminotransferase, lactate dehydrogenase, creatine kinase, and creatine kinase isoenzymes. According to the data in Figure 9, there is no significant difference between the experimental group and the control group in the levels of myocardial enzymes before the experiment. After the experiment, the levels of myocardial enzymes in the two groups dropped significantly, but according to the chart range, the levels of myocardial enzymes after professional care dropped more significantly. It shows that the recovery effect of the experimental group is better.

### 4.3. Postoperative Analysis of Patients with Acute Myocardial Infarction

According to the data in Figure 10, the postoperative conditions of patients with acute myocardial infarction are the same. Cardiovascular and cerebrovascular accident is a common disease that seriously threatens the health of human beings, especially the middle-aged and elderly people over 50 years old. Even with the most advanced and complete treatment methods, more than 50% of cerebrovascular accident survivors cannot fully take care of themselves. In terms of the recovery of cardiovascular and cerebrovascular, according to the histogram, it can be seen that the recovery degree of the control group in the first two months is due to the experimental group, but the gap is very small. In the third month of guidance, the recovery status of the experimental group began to surpass that of the control group, and the gap continued to widen in the subsequent months of recovery, indicating that postoperative scientific care is necessary. From the analysis of mortality, the conditions of the two groups of experimental patients are the same, but the mortality rate of patients in the control group is higher than that of the experimental group, especially in the first month after surgery, and the gap between the two experiments is very large. In summary, carrying out scientific and effective care can improve the survival rate of patients.

RETRACTED

## 5. Conclusions

First aid is the meaning of emergency treatment, which means that when any accident or emergency occurs, the rescuer, before the arrival of the medical staff, according to the principle of medical care, temporarily and appropriately conducts preliminary rescue and treatment for the wounded and sick by using the materials available on site. In the context of medical treatment, this article is combined with the current developing economy. The purpose is to study the effect of a stratified emergency care team assisted by multidisciplinary first aid knowledge in the first aid of acute myocardial infarction, hoping to reduce the probability of acute myocardial infarction through first aid and nursing. In this paper, the BPR theory is used to construct the AMI emergency care process in the hospital, which effectively reduces the emergency delay time of AMI patients, improves the patient's emergency response, and improves the efficiency of emergency nurses' rescue work. Overall, the following tasks are mainly completed: (1) the calculation knowledge of medical image registration is introduced, its evolution process is introduced in detail, and the image conversion process is briefly explained. (2) The relevant knowledge of emergency medicine was collected and sorted, and the necessary database was established to save time for the emergency process. (3) After measuring the energy consumption of the preliminary plan, the exercise rehabilitation plan for patients after acute myocardial infarction is finally formed, which provides a blueprint for the timely rehabilitation of patients.

## Figures and Tables

**Figure 1:** Schematic diagram of myocardial infarction.

**Figure 2:** Principle of spatial transformation.

**Figure 3:** Image conversion process.

**Figure 4:** Schematic diagram of the geometric transformation.

**Figure 5:** Structure of the knowledge system.

**Figure 6:** Treatment status of patients with acute myocardial infarction.

**Figure 7:** Cardiac function status of patients with acute myocardial infarction.

RETRACTED

**Figure 8:** Treatment results for the two groups of patients.

**Figure 9:** Comparative analysis of cardiac enzyme profiles before and after treatment.

**Figure 10:** Analysis of postoperative conditions in patients with acute myocardial infarction.

**Table 1:** Basic patient information.

Variables	1	2	Average
Age	66	67	66.5
Male	300	300	300
Blood pressure	130	150	140
Diabetes	200	180	190
Medical history	15	9	12

**Table 2:** Comparison of patient rescue times.

Variables	1	2	Average
Percutaneous coronary intervention	210	220	215
Emergency percutaneous coronary intervention	180	150	165
SO-to-B (min)	430	440	435
SO-to-FMC (min)	250	250	250
FMC-to-B (min)	150	160	155
SO-to-D (min)	330	350	340

**Table 3:** Number of branches of diseased vessels in patients with myocardial infarction.

	ST-segment elevation myocardial infarction	Non-ST-segment elevation myocardial infarction	Total
Negative	1	0	1
Single branch	240	90	330
Double	45	130	175
Multiple	7	40	47

**Table 4:** ECG status in patients with acute myocardial infarction.

Electrocardiographic features	Sensitivity (%)	Specificity (%)
ST↓aVLI	80	89.2
STV3 ↓ /STIII↑≤1.2	75.3	82.7
STI ↓ ≥0.05 mV	60.3	65.2
ST↑III > II	82.1	82.1

## Data Availability

This article does not cover data research. No data were used to support this study.

## References

[1] Noris P., Bertolino G., Previtali M., Ferrario M., Balduini C. L. (2004). Heparin infusion facilitates ex vivo spontaneous platelet aggregation in patients with acute myocardial infarction who have undergone thrombolytic therapy. *Pathophysiology of Haemostasis and Thrombosis*.

[2] Eicher J. D., Wakabayashi Y., Vitseva O. (2016). Characterization of the platelet transcriptome by RNA sequencing in patients with acute myocardial infarction. *Platelets*.

[3] Shah R. U., de Lemos J. A., Wang T. Y. (2016). Post-hospital outcomes of patients with acute myocardial infarction with cardiogenic shock: findings from the NCDR. *Journal of the American College of Cardiology*.

[4] Avau B., Vande veegaete A., Scheers H., Vandekerckhove P., de Buck E. (2019). Determining first aid knowledge and skills retention with laypeople: a randomized controlled trial in Nepal. *International Journal of First Aid Education*.

[5] Qing Y., Yongqiang X., Xiaoming F. (2020). First-aid knowledge regarding small area burns in children among 5814 caregivers: a questionnaire analysis. *Burns*.

[6] Zhang Q., Qi W., Yao W., Wang M., Chen Y., Zhou Y. (2016). Ambient particulate matter (PM2.5/PM10) exposure and emergency department visits for acute myocardial infarction in Chaoyang District, Beijing, China During 2016: a case-crossover study. *Journal of Epidemiology*.

RETRACTED

[7] Zhang H., Song D., An L. (2016). Effect of a real-time tele-transmission system of 12-lead electrocardiogram on the first-aid for athletes with ST-elevation myocardial infarction. *Pakistan Journal of Pharmaceutical Sciences*.

[8] Gopinath G., Gv K. G., Sasikumar H., Tamilanban Y., Patil J., Gopinath G. (2021). A novel artificial intelligence based Internet of Things for fall detection of elderly care monitoring. *Journal of Intelligent Systems and Internet of Things*.

[9] Luiz T., Dittrich S., Pollach G., Madler C. (2017). Knowledge of the population about leading symptoms of cardiovascular emergencies and the responsibility and accessibility of medical facilities in emergencies: results of the KZEN study in Western Palatinate. *Der Anaesthesist*.

[10] Al-Dubai S., Aas A., Sabori S. (2018). Knowledge and practice of first aid among parents attending primary health care centers in Madinah City, Saudi Arabia, a cross sectional study. *Journal of Family Medicine and Primary Care*.

[11] Pei L., Liang F., Sun S., Wang H., Dou H. (2019). Nursing students' knowledge, willingness, and attitudes toward the first aid behavior as bystanders in traffic accident trauma: a cross-sectional survey. *International Journal of Nursing Sciences*.

[12] Alkhotani A. M., Almalki W. M., Alkhotani A. M., Turkistani M. A. (2019). Makkah female teachers' knowledge of seizure first aid. *Epilepsy & Behavior*.

[13] Luckie K., Pang T. C., Kritikos V., Saini B., Moles R. J. (2018). Development and validation of an asthma first aid knowledge questionnaire. *Research in Social and Administrative Pharmacy*.

[14] Yu Q., Xiao Y. Q., Hu X. Y., Xia Z. F. (2019). Cognitive level of first aid knowledge regarding small area burn among 2 723 child caregivers in Shanghai: a cross-sectional survey and analysis. *Zhonghua shao shang za zhi = Zhonghua shaoshang zazhi = Chinese journal of burns*.

[15] Schiefer J. L., Schuller H., Fuchs P. C. (2020). Burn first aid knowledge in Germany and the influences of social-economic factors. *Burns*.

[16] Ibrahim A., Sam-Agudu N., Omaye U., Ushie B., Olumide A., Omotade O. (2016). 933Impact of first aid training on the first aid knowledge and skills capacity of primary school teachers in Ibadan, Nigeria. *Injury Prevention*.

[17] Iyer S. S., Panigrahi A., Sharma S. (2017). Knowledge and awareness of first aid of avulsed tooth among physicians and nurses of hospital emergency department. *Journal of Pharmacy & Bioallied Sciences*.

[18] Baginska J., Rodakowska E., Milewski R., Wilczynska-Borawska M., Kierklo A. (2016). Polish school nurses' knowledge of the first-aid in tooth avulsion of permanent teeth. *BMC Oral Health*.

RETRACTED

[19] McNamara R. L., Kennedy K. F., Cohen D. J. (2016). Predicting in-hospital mortality in patients with acute myocardial infarction. *Journal of the American College of Cardiology*.

[20] Chapman A. R., Anand A., Boeddinghaus J. (2017). Comparison of the efficacy and safety of early rule-out pathways for acute myocardial infarction. *Circulation*.

[21] Caretti G., Berghella L., Juan A., Latella L., Ryall J. (2016). Epigenetic regulation shapes the stem cells state. *Stem Cells International*.

[22] Dondo T. B., Hall M., West R. M. (2017). *β*-blockers and mortality after acute myocardial infarction in patients without heart failure or ventricular dysfunction. *Journal of the American College of Cardiology*.

[23] Berliner T. (2018). Oxygen therapy in suspected acute myocardial infarction: Hofmann R, James SK, Jernberg T, et al. N Engl J Med. 377; 13: 1240-1249. *Journal of Emergency Medicine*.

[24] Hofmann R., James S. K., Jernberg T. (2017). Oxygen therapy in suspected acute myocardial infarction. *New England Journal of Medicine*.

[25] Thiele H., Akin I., Sandri M. (2017). PCI strategies in patients with acute myocardial infarction and cardiogenic shock. *New England Journal of Medicine*.

[26] Noguchi T., Yasuda S., Shibata T. (2016). Response to letter regarding article, "prevalence, clinical features, and prognosis of acute myocardial infarction attributable to coronary artery embolism". *Circulation*.

[27] Lancet T. (2016). Acute myocardial infarction in women. *Lancet*.

[28] Westman P. C., Lipinski M. J., Luger D. (2016). Inflammation as a driver of adverse left ventricular remodeling after acute myocardial infarction. *Journal of the American College of Cardiology*.

[29] Carlo D. M., Mara S., Flavio A. (2016). Single vs multivessel treatment during primary angioplasty: results of the multicentre randomised HEpacoat for cu LPrit or multivessel stenting for acute myocardial infarction (HELP AMI) study. *International Journal of Cardiovascular Interventions*.

[30] Krichen M., Mechti S., Alroobaea R. (2021). A formal testing model for operating room control system using internet of things. *Computers, Materials & Continua*.

[31] Talebi A., Bodagh M., Falahi B. (2020). Investigation of the effect of ACT-SMART on nurses' perceived level of violence management in emergency section. *Preventive Care In Nursing and Midwifery Journal*.

[32] Cho G. Y. (2016). Effects of a simulation-based education on cardiopulmonary emergency care knowledge, critical thinking and problem solving ability in nursing students. *Journal of Fisheries and Marine Sciences Education*.

[33] Tabassum K., Shaiba H., Essa N. A., Elbadie H. A. (2022). An efficient emergency patient monitoring based on Mobile ad hoc networks. *Journal of Organizational and End User*.

